This article has been retracted.

# Discussion on Basic Japanese Teaching Mode in Multimedia Network Environment

**DOI:** 10.1155/2022/7797540

**Published:** 2022-07-15

**Authors:** JianXue Xia

**Affiliations:** Foreign Languages School, Nanyang Normal University Nanyang, Nanyang, Henan 473000, China

## Abstract

With the development of the information age and the progress of science and technology, the traditional education model cannot meet the needs of teachers and students for richer knowledge and diversified teaching methods in the new era. The traditional basic Japanese teaching mode has not matched with the current form of social development. Therefore, it is urgent to establish a new basic Japanese teaching model. The development of multimedia brings the Internet mixed teaching mode, which just fills the gap of this kind of teaching method and provides new ideas and ways for the reform of teaching methods. The application of multimedia network assisted teaching in basic Japanese teaching plays a great role in promoting basic Japanese teaching. In the multimedia network environment, how to let students learn independently, find and raise problems by themselves, and analyze and solve problems at a deeper level has attracted the attention of many educators. Improving the practicability of Japanese teaching is very important for Japanese teaching in colleges and universities. Therefore, this paper studies media teaching, analyzes the current and existing problems of multimedia teaching in Japanese teaching and the principles that should be followed in order to develop, finds the limitations of using multimedia teaching methods in the current Japanese teaching and learning process, and puts forward targeted suggestions and application strategies on these limitations, and builds a new model of basic Japanese teaching under the multimedia network environment.

## 1. Introduction

In the context of the rapid development of information, multimedia and network technologies have been widely used in foreign language teaching [1]. In basic Japanese teaching, the traditional teaching mode can no longer meet the social demand for high-quality innovative Japanese talents. Under the traditional education mode, the main body in the classroom is teachers, students are in a passive position, and the way of knowledge reception belongs to indoctrination. Therefore, it is urgent to establish a new basic Japanese teaching model [2]. The use of multimedia network-assisted teaching in basic Japanese teaching has a great role in promoting basic Japanese teaching, but there are also some shortcomings [3]. It is an important issue that basic Japanese teachers must solve to explore a set of effective new models of basic Japanese teaching [4].

At present, with the continuous development of information technology, all kinds of intelligent devices extended by multimedia have basically been popularized in the daily life of the public [5]. The emergence of information technology not only brings great convenience to the public's daily life but also plays an important role in the field of education. Under the Internet online education mode, teachers and students can use the Internet to complete the two links of teaching and learning with the support of information technology means when they are not in the same space. Teachers' teaching methods are more novel, teaching priorities are more prominent, and students' learning process is more active, so the educational effect is more remarkable. In this context, Chinese universities have also introduced the teaching mode of “multimedia + education” in Japanese teaching [6]. Among them, Japanese MOOCs, microcourses and other forms are hybrid teaching modes, which have become indispensable for many colleges and universities to carry out teaching work [7]. How to give full play to the active role of Japanese blended teaching under the background of “multimedia + education” and promote the organic combination of multimedia carriers and traditional teaching has become an important issue in college education today [8]. The mixed teaching mode not only improves students' enthusiasm in Japanese learning but also enhances the interaction between teachers and students, so as to enrich the Japanese teaching content and optimize the teaching effect. Therefore, it is very important for the development of China's education to study how to carry out Japanese online teaching and ensure the quality of Japanese teaching.

## 2. The Current Situation and Trend of Using Multimedia and Network-Assisted Teaching in Basic Japanese Teaching

The basic stage of Japanese learning is the most important link in the process of Japanese learning. However, due to the limitations of traditional Japanese teaching habits and teaching concepts, Japanese teaching is often based on grammar translation method and measured by examination results. It only pays attention to the mechanical learning of language and ignores the purpose of communication and communication in professional Japanese teaching [9]. This will inevitably lead to teachers playing a leading role in teaching. They pay too much attention to the teaching of basic knowledge such as grammar, and often neglect the cultivation of students' application ability and communicative ability [10]. With the continuous increase of the number of Japanese majors and the increasingly severe employment situation, the traditional basic Japanese teaching mode has been difficult to adapt for the development of the social situation [11].

With the development of modern educational technology, multimedia and network-assisted teaching have been widely used in foreign language teaching. Multimedia network teaching refers to the application of multimedia and network technology to collect, transmit, process and share educational and teaching resources, and use computers to achieve teaching goals [12]. Multimedia network teaching is a new teaching method that combines traditional teaching with modern multimedia network technology. It provides a visual teaching environment that is easy for collaborative learning. Under the influence and promotion of the general environment, more and more Japanese teachers begin to use multimedia network to assist teaching. In basic Japanese teaching, multimedia network-assisted teaching has been widely popularized and has become a trend [13].

At present, most Japanese teachers in colleges and universities have adopted multimedia network-assisted teaching [14]. In basic Japanese teaching, teachers mainly use multimedia network technology, with the help of words, sounds, images, images, etc., through courseware to convert abstract words, grammar, texts, etc. The learning provides rich teaching scenarios [15]. Under the stimulation of various senses, students are deeply impressed by the Japanese knowledge they have learned, and through the imitation and practice of Japanese original sound and Japanese scenes, students can arouse their strong interest in learning, enhance students' learning effect, and achieve the purpose of Japanese learning [16]. In recent years, Japanese teachers in many colleges and universities, especially young Japanese teachers, have not only turned rich network resources into teaching materials in basic Japanese teaching but also opened up a second classroom through network means such as emails, forums, and chat tools, broadening the students' study space providing more learning opportunities for students [17].

The goal of carrying out the Japanese blended teaching reform is not only to improve the content of Japanese teaching in colleges and universities but also to stimulate students' interest in learning and improving students' Japanese communication level as shown in Table 1. However, at present, in the process of Japanese blended teaching in some colleges and universities, there have been problems such as insufficient preclass design, insufficient classroom process, and imperfect after-class evaluation, which will affect the improvement of students' learning ability in the long run. Therefore, college teachers are needed. Analyze it in depth [18]. In the future, multimedia education and teaching will be more “intelligent” in the network environment. For example, with the support of algorithm technology, teachers can use computer database to record students' learning progress and recent learning situation. Through data planning, teachers can adjust their own teaching scheme according to students' weaknesses, so as to carry out personalized training.

## 3. Teaching Advantages of Japanese Mixed Course in Multimedia Network Environment

With the increasing frequency of international exchanges, my country needs more high-quality language talents to fill the social gap. Colleges and universities, as the main front of talent training, have seen a marked improvement in the overall situation of education and teaching in recent years under the guidance of the goals of education and teaching reform [19]. Taking Japanese blended teaching as an example, the combination of multimedia and Japanese teaching in colleges and universities, and the use of blended teaching mode can greatly enhance students' understanding of Japanese, improve teaching quality, and realize teaching reform. Therefore, studying the combination of the two has certain teaching advantages as shown in Figure 1.

### 3.1. Massive Online Textbook Resources

Under the background of big data, the rational use of blended teaching mode in Japanese language course teaching in colleges and universities can accumulate rich teaching resources. For example, our school requires students to take the CET-4 for College Japanese, which has relatively high requirements for students' reading ability, but the teaching materials are simple in content and less in length, which is far from the requirements of the test. Using blended teaching, students can download reading materials of different levels of difficulty from the Internet for reading after class. While improving the reading quality, they can also accumulate good words and sentences, and accumulate materials for the word-building and sentence-building part of the test. When preparing teaching courseware, teachers can not only find Japanese chapters suitable for students' learning difficulty on the Internet but also download classroom videos and teaching courseware of other famous teachers in colleges and universities.

### 3.2. Three-Dimensional Teaching Environment

Three-dimensional intelligent teaching environment “Multimedia + Japanese” teaching is a model that combines traditional classroom teaching with intelligent Japanese teaching, which can fully create a three-dimensional teaching environment and stimulate students' interest in learning. For example, teachers play Japanese teaching videos with the help of information technology, carry out situational teaching, and encourage students to actively participate in classroom interaction. In addition, teachers can use information technology to conduct simultaneous translation, role dubbing, online live teaching and other rich teaching links with students, so that students can efficiently complete their learning tasks.

### 3.3. Multi-Information Teaching Mode

The development of the Japanese hybrid teaching mode in colleges and universities can effectively integrate various teaching modes such as MOOCs, microcourses, cloud classrooms, and project-based teaching, and maximize the enrichment of information-based teaching methods. For example, teachers can use the shared screen to conduct live teaching through Tencent Classroom or video conferencing functions. After the course is over, the system can automatically save the teaching content of this course to form a teaching video. Students can learn repeatedly after class to consolidate what they have learned in class. In addition, teachers can also arrange project-based teaching tasks offline. Students use video production, learning recording, etc. to complete homework and upload it to the teaching platform, which greatly saves teaching time in offline classrooms, making Japanese teaching convenient and efficient.

### 3.4. The Role of Multimedia Network Technology in Promoting Basic Japanese Teaching

Most Japanese majors choose Japanese as a major because they have a strong interest in Japanese. The author once conducted a survey on freshmen from grade 07 to grade 11 in a school, and more than half of the students in each class chose Japanese because they were interested in Japanese animation. Therefore, basic Japanese teachers can combine this actual situation in teaching, change the traditional monotonous teaching method centered on text and grammar, make full use of multimedia network-assisted teaching, and organically combine text, sound, animation, etc. The teaching is lively and interesting, allowing students to easily master basic Japanese knowledge in a close-to-real scene, and stimulate and improve students' interest in learning Japanese as shown in Figure 2.

The teaching content of the basic stage of Japanese majors mainly includes six items:

This not only allows students to master the basic knowledge of Japanese such as vocabulary and grammar but also cultivates students' basic skills in listening, speaking, reading and writing, and also cultivates the ability to practically apply the language as shown in Figure 3. According to the actual situation of students, through multimedia network technology, rich network resources are used to supplement the teaching content, so that students can come into contact with a large number of Japanese original sounds and real scenes both inside and outside the classroom. Teachers train students in listening, speaking, reading and writing through selected materials, and appropriately explain grammar and sentence patterns in combination with texts and background materials, so that students can exercise and improve listening skills on the basis of mastering vocabulary, grammar, sentence patterns and other meanings, speaking, reading, writing, translation and other comprehensive ability. In addition, teachers make full use of network resources to carry out various teaching activities, such as organizing students to focus on the texts they have learned, and select appropriate network resources for question and answer, retelling, performance, discussion, publication, etc., which can not only deepen students' understanding of the text but also help to improve students' Japanese application ability and communication ability.

Through multimedia network-assisted teaching, teachers make full use of network resources, and can select listening, reading, video and other materials with moderate content difficulty and recommend them to students through e-mail and other network means according to the teaching progress and the actual situation of students, so as to open up students' learning space. Through the multimedia network, students can repeatedly practice the content that they have not mastered in class after class, and can also conduct personalized learning according to their own situation. Teachers can also guide students to make good use of Japanese learning websites, Japanese electronic newspapers and periodicals, online libraries, dictionaries, etc., to exercise and cultivate students' self-learning ability. In the process of mutual integration of information technology and Japanese course teaching, teachers can reasonably design preclass preview links, in class interaction links and after-school reflection links for students through the combination of online teaching and offline teaching, and improve students' learning autonomy and learning ability through interaction and communication with students. At the same time, it can also help students explore and learn online and improve their learning level. In addition, under the background of “Internet +,” rebuilding the Japanese teaching mode can also improve students' classroom interaction and communication ability, so that students can truly become the masters of classroom learning. Moreover, through mobile learning or visual learning, students can improve their ability to master knowledge points.

From the above analysis, it can be seen that teachers' use of multimedia network-assisted teaching in basic Japanese teaching can make up for the deficiencies of traditional teaching methods and lay a solid foundation for Japanese learning in senior grades.

## 4. Disadvantages and Shortcomings of Using Multimedia and Network Technology in Basic Japanese Teaching

### 4.1. Teachers' Use of Multimedia Network Technology in Basic Japanese Teaching Is often Limited by Computer Application Ability

Although it has become a trend to use multimedia network to teach Japanese, due to the limitation of technical level, some teachers, especially middle-aged and elderly teachers, are not good at the application of computer and network technology, and cannot use multimedia network technology to basic Japanese with ease as shown in Figure 4. There are many teachers who cannot concentrate on teaching itself. The author has conducted research on the basic Japanese teaching situation in some domestic colleges and universities. The basic Japanese teachers in most colleges and universities have adopted multimedia network-assisted teaching to varying degrees, but some basically still use the traditional teaching mode of “one blackboard and one chalk.” Mainly, the multimedia teaching system is just a decoration. Although some also have courseware, the content is monotonous and empty, and it does not play any role at all, let alone protect the interest of students.

### 4.2. The Use of Multimedia Network-Assisted Teaching in Basic Japanese Teaching Is Also Limited by Some Objective Conditions

Having a complete set of multimedia teaching system is a prerequisite for teachers to make full use of multimedia network-assisted teaching. Today, almost all colleges and universities are equipped with multimedia teaching systems, but the quality of equipment varies. Some multimedia teaching facilities with poor quality will have problems such as no sound or unclear sound, unclear images, etc., which will inevitably affect the teaching effect more or less. Even a well-equipped multimedia teaching system is sometimes affected by objective factors such as power outages, network interruptions, and network speeds. Such objective factors often lead to the failure to play the courseware carefully crafted by teachers, and students will be unable to access the Japanese original sound or real scenes in the classroom, which will naturally have a certain impact on the effect of the class. Also, not all students have a computer in hand. Especially freshmen who have just entered the school, not many are equipped with computers in the first semester. Therefore, when basic Japanese teachers forward some learning materials to students through the Internet, they should consider objective factors such as whether students are equipped with computers and whether they have access to the Internet.

### 4.3. Excessive Use of Multimedia Network-Assisted Teaching in Basic Japanese Teaching Often Affects the Effect of Teaching and Learning

Confucius said: “Too much is too much.” In basic Japanese teaching, too much use of multimedia technology and too much use of network resources is not a good thing. For example, for first-year freshmen, teachers use multimedia network to assist teaching too much from the beginning, and students will have varying degrees of dependence on multimedia courseware. The author once observed students in a class and found that very few students took notes. Even though the importance of taking notes has been emphasized many times, there are still many students who are reluctant to take notes, and their memory of knowledge flashes with the slides. If the memory is not good, and there is no review and consolidation after class, the students' learning effect can be imagined. In basic Japanese teaching, too much use of multimedia and too much use of network resources not only wastes a lot of time for teachers to collect and organize a large number of teaching materials but also the seemingly fancy courseware cannot make students achieve the desired learning effect. In addition, because students have a strong dependence on courseware, they will be full of expectations for the teacher's courseware. If the teacher's courseware in this lesson is not as exciting as the previous lesson, it will be difficult for some students to arouse their interest, which will affect the students' learning effect. In addition, excessive use of multimedia network to assist teaching will also cause students to ignore the role of teachers. In traditional basic Japanese teaching, teachers dominate. In the multimedia network environment, students can use the rich network resources by themselves, come into contact with a large number of Japanese materials and Japanese learning environment, and can carry out selective and targeted self-study according to their own interests and needs. Even in basic Japanese classes, there is often too much emphasis on the content of the teacher's courseware, while ignoring what the teacher says when playing the courseware. What is more, some students have some knowledge of what they have learned in advance through the Internet. When the teacher talks about this knowledge in class, some students no longer listen carefully to the teacher's explanation, even if some students only know a little. Over time, students will feel that the role of the teacher is not important.

It can be seen that basic Japanese teachers should be proficient in computer and network technology. When using multimedia network to assist teaching, we should not use multimedia technology and network resources too much, nor should we make students rely on multimedia and network, thus ignoring the role of teachers.

Make full use of the preclass preparation stage For Japanese teaching in colleges and universities, teachers should pay attention to the use of preclass preparation design time in the process of carrying out blended teaching, help students to do preclass knowledge guidance, and clarify the learning direction of this class. Teachers can prepare a learning task list in advance, combine the content of the course, make a tutorial plan through video or animation, and intersperse chapter practice questions and test questions in it, requiring students to complete it before class, so that students can enjoy a relaxed and happy atmosphere. Complete the preclass preparation and be fully prepared for the class.

Do a good job in the implementation and planning of teaching courses teaching courses are the core of Japanese blended teaching. Only in the classroom can students fully interact with teachers and master Japanese grammar and word formation rules. Specifically: Teachers can integrate micro-lectures, video design and teaching interaction in the class, organize and upload knowledge points to the cloud teaching platform, collect common problems in a centralized manner, and use various methods to solve them in the classroom in a timely manner. For example, in the difficult part of honorifics in Japanese teaching, teachers can first collect feedback from students through preclass preview, set up a storyline for students, and compare the differences between honorifics, self-effacing and solemn expressions in Japanese with sentence pattern rules Translate and explain word by word, and then ask several students to have a dialogue according to the video instructions, or design sketches to imitate performances, so as to help students master the knowledge points in the class and complete the construction of the knowledge system in the blended learning.

## 5. Building a New Mode of Basic Japanese Teaching in the Multimedia Network Environment

### 5.1. Effective Combination of Traditional Teaching Mode and Multimedia Network-Assisted Teaching

Basic Japanese teachers should keep up with the pace of the times, pay attention to the updating of their own knowledge, and continuously improve their computer and network application capabilities as shown in Table 2. In the teaching process, we should realize the effective combination of traditional teaching mode and multimedia network assisted teaching according to the teaching objectives and teaching contents, combined with the actual situation of students. For example, although there are a large number of Chinese characters in Japanese, the writing of some Japanese characters is very different from that of Chinese characters. Only by showing and emphasizing them in the courseware cannot make Japanese beginners truly grasp the difference between Japanese characters and Chinese characters. When it is necessary to emphasize these Chinese characters, teachers can use chalk to write their stroke order, radicals, etc., on the blackboard one by one. Only by witnessing the teacher's writing process can students remember the writing of these Chinese characters. There will be no errors during use. It can be seen that today's multimedia network-assisted teaching has become popular, but the traditional “one blackboard, one chalk” cannot be discarded. Of course, while using the traditional teaching mode to impart knowledge to students, teachers can also combine multimedia network-assisted teaching to further strengthen the effect of classroom teaching. Japanese words are taken that are similar to Chinese characters but have different meanings as an example. When basic Japanese teachers teach vocabulary containing these Chinese characters, they use the traditional teaching mode to let students master the writing of these Japanese characters, and then they can use multimedia. Network-assisted teaching allows students to further understand the pronunciation, meaning and usage of these Chinese characters, and can also expose students to pictures, texts, Japanese soundtracks and real scenes containing these Chinese characters as needed. In this way, teachers can achieve good teaching effect only by effectively combining traditional teaching mode with multimedia network-assisted teaching. Students can also master basic knowledge in a relaxed atmosphere, and improve their listening, speaking, reading, writing, translation and other abilities, and achieve good learning results.

### 5.2. Grasp the “Degree” of Using Multimedia Network-Assisted Teaching

Today, with the rapid development of information and the popularization of multimedia network-assisted teaching, rich network resources do provide a lot of materials for Japanese learning, but the proliferation of network resources also leads to a large number of Japanese materials that are disorganized and lack systematization and integrity. Although the traditional paper textbooks have a certain lag, they are often carefully selected, and the systematicness and integrity of their knowledge structure are unmatched by network resources. Therefore, teachers should avoid excessive use of network resources and ignore the textbook itself in basic Japanese teaching. When teachers use multimedia technology in basic Japanese teaching, they must adhere to the principles of science and rationality, grasp the “degree” of using multimedia network-assisted teaching, and try to avoid too much attention to the form of courseware and dependence on courseware. When making multimedia courseware, teachers strive to be concise and clear, and highlight the key points and difficulties, so as to avoid distracting students' attention due to too fancy courseware, and avoid excessive content of courseware affecting students' learning effect.

### 5.3. Teachers Play an Active Guiding Role and Create a Japanese Teaching Situation

Since most of the students majoring in Japanese start learning Japanese from scratch, basic Japanese teachers have an important responsibility and must actively guide students so that they can firmly grasp the basic knowledge as shown in Table 3. Teachers can make full use of modern information technology such as multimedia technology as an aid. Realistic teaching situations can stimulate students' imagination, make students feel as if they are really in the actual scene, and promote students to more deeply understand the content of Japanese language knowledge in the situation. Teachers can design many situations for students to solve the same problem through multimedia videos, so that students can understand the same knowledge point from multiple angles. This is not only conducive for the improvement of students' Japanese knowledge structure but also has a very positive significance for the improvement of students' Japanese practical ability. When using multimedia technology, teachers can fully mobilize students' classroom enthusiasm, so that students can better experience the situation and feel a more realistic and rich Japanese language environment. In such an environment, students' language perception ability will be well cultivated, and with the improvement of language perception ability, their cultural understanding and language application ability will be gradually improved, which will drive the overall teaching quality of comprehensive Japanese.

### 5.4. Establish and Improve the Network Implementation Platform for Basic Japanese Teaching

On the basis of the Internet, the online teaching platform provides comprehensive support for the implementation of online teaching. At present, many colleges and universities have used the Blackboard online teaching platform, which integrates the functions of curriculum development, online teaching, and teaching resource management. Basic Japanese teachers can establish and improve the online teaching implementation platform of basic Japanese courses according to their needs, upload teaching materials, publish course information, conduct online tests or teacher-student discussions through the platform, and transform the closed basic Japanese teaching into an open basis Japanese teaching provides students with a platform for independent learning, and uses multimedia network technology to monitor and evaluate students' learning intelligently.

### 5.5. Problems That Should Be Paid Attention to in the Application of Multimedia Methods in College Japanese Teaching

As a typical representative of modern teaching methods, multimedia teaching must abandon the traditional “cramming” or “indoctrination” of outdated teaching ideas, and put an end to the emergence of the new “cramming” teaching phenomenon of “speaking on the screen” as shown in Figure 5. Human beings invented language in order to better carry out communication. Professional Japanese teaching serves for better communication. At present, many college teachers still stay in the classroom in Japanese teaching and do not really apply the law of learning and mastering the language. This is also a place where the construction of College Japanese major should be focused and solved. Only by putting the language in its inherent place, learning and mastering the language can we really join the society. Under the brand-new college Japanese teaching method, teachers must be freed from the mechanical teaching of backward grammar, and vocabulary truly plays the role of “assistant” in teaching and establishing modern teaching ideas. At the same time, students should also get rid of the traditional purely passive learning concept, establish an active learning idea, actively participate in the whole teaching process, and improve their own consciousness, purpose and initiative in Japanese learning.

Under the guidance of the country's policy of vigorously calling for the use of new technology in teaching, many Japanese teachers in colleges and universities have used multimedia teaching in order to use multimedia teaching, that is, pure formalism. This situation not only fails to give full play to the advantages and functions of multimedia teaching methods but also seriously hinders college students' learning and mastering of Japanese knowledge. Therefore, the majority of Japanese teachers in colleges and universities should establish a correct concept of multimedia teaching, carefully prepare each courseware, try to eliminate some irrelevant knowledge content, pictures, sounds or special effects, etc., avoid the occurrence of any formalism, and realize multimedia methods in college Japanese. The maximization of function and value in teaching will promote the sustainable and healthy development of Japanese language teaching in Chinese universities.

The application of multimedia teaching methods in college Japanese teaching is not a complete replacement of the traditional teaching mode. Although the multimedia teaching method has many advantages and characteristics, the traditional teaching mode still has its own unique teaching function and value. For the current college Japanese teaching, whether it is simply adopting multimedia teaching methods or simply using traditional teaching models, it is impossible to optimize the effect of college Japanese teaching. Only the scientific and rational combination of multimedia teaching and traditional teaching mode can promote the highest quality of Japanese teaching in colleges. Specifically, for some highly communicative knowledge points, they can be explained through multimedia video demonstrations, so as to promote students' comprehensive understanding and mastery of pronunciation, words, expressions, body movements, etc.; explanation or vocabulary with unique usage, etc., can deepen the impression of students through blackboard writing. The combination of multimedia teaching methods and traditional teaching modes can make up for each other's shortcomings to the greatest extent, so as to truly improve the teaching effect of college Japanese.

## 6. Conclusion

In the “Internet +” era, the way of information acquisition has been changed, the time and space constraints have been broken through, and the traditional Japanese teaching mode in colleges and universities is also facing reform and innovation. Under the trend of integrating the traditional teaching mode with the application of Internet technology, teachers no longer need to integrate the traditional teaching mode into the traditional teaching system. Give full play to the guiding role of teachers, stimulate students' initiative, build an open, equal, interactive and independent Japanese learning classroom for students, and perfectly combine teaching and learning. At the current stage, many colleges and universities have integrated the model of “multimedia + education” into Japanese teaching, forming a new hybrid teaching model, which not only enriches the content of Japanese teaching but also promotes the reform of Japanese professional teaching and cultivates high-quality language for the society. In recent years, through the analysis and research on the reform of Japanese course teaching in colleges and universities, it can be seen that information teaching is not only the requirement of the times but also the inevitable result of the educational situation. Therefore, in the process of Japanese mixed teaching, teachers need to pay attention to the integration and use of online and offline resources, summarize the problems and deficiencies in teaching in a timely manner, and provide more valuable teaching experience for the reform of Japanese teaching, thereby improving the quality of Japanese teaching.

The use of multimedia network assisted instruction in basic Japanese teaching can make up for the shortcomings of traditional teaching methods and greatly promote basic Japanese teaching, but there are also some problems, such as old views, insufficient equipment, formalism and so on. Basic Japanese teaching has a long way to go. In the process of building a new mode of basic Japanese teaching in the multimedia network environment, basic Japanese teachers must adhere to the effective combination of traditional teaching mode and multimedia network-assisted teaching, and constantly improve teaching methods and teaching methods. Put forward effective measures for basic Japanese teaching reform to maximize the effect of basic Japanese teaching.

## Figures and Tables

**Figure 1:** Teaching advantages of Japanese mixed course in multimedia network environment.

**Figure 2:** The role of multimedia network technology in promoting basic Japanese teaching.

**Figure 3:** Six items of teaching content in the basic stage of Japanese majors.

**Figure 4:** Disadvantages and shortcomings of using multimedia and network technology in basic Japanese teaching.

**Figure 5:** Problems that should be paid attention to in the application of multimedia methods to college Japanese teaching.

**Table 1:** Current situation of Japanese mixed course teaching under the multimedia + background.

1	Preclass design teaching is not enough in the Japanese blended teaching model, but preclass design is a very important part. Some students can take notes, data query, phrase translation and other work in advance according to the teacher's preclass design guidelines, so as to improve the classroom teaching efficiency. However, some colleges and universities do not pay enough attention to preclass teaching design and after-class teaching design. The progress of preclass preview and chapter preview is not checked and supervised in time, and students are not required to complete online preclass homework on time. The quality of the prepreparation is not high, which greatly affects the development of the teaching plan in class

2	The content of blended teaching is not rich enough in the process of Japanese blended teaching in some colleges and universities, and the teaching content in class is not rich enough. Teachers simply use information technology to show teaching courseware and teaching videos, and seldom use information media to interact with students, which fails to fundamentally change the passive learning situation of students, which makes it difficult for students to understand and build sentence thinking frameworks in the teaching section of reading and writing. For example, in the face of the requirements of the four-level grammar and word formation and sentence construction of college Japanese, students need to understand the difference between Chinese and Japanese grammar, and have a firm grasp of Japanese grammar. Some teachers only show students relevant teaching video analysis, practical practice sessions and tests. There are few links, resulting in insufficient output of students, and the practical application ability of grammar cannot meet the test requirements

3	The teaching evaluation link is relatively simple. At present, in some colleges and universities, after-school teaching evaluation is often easily ignored. Although some colleges and universities will regularly carry out teaching evaluation content and organize students to use paper version or computer platform to conduct teaching evaluation, the formalization in the actual operation process is more obvious, so most of the suggestions made are irrelevant and miss the point. In addition, when some teachers carry out the teaching self-evaluation link, it is mostly because of the apparent problem that the integration of information technology is not deep enough, and they are unable to deeply reflect and evaluate the root cause of teaching. In addition, the teaching evaluation only adopts simple teaching evaluation methods such as student evaluation and teacher evaluation, and the form is single, which is difficult to meet the teaching needs.

**Table 2:** A new mode of basic Japanese teaching under the construction of multimedia network environment.

1	Effective combination of traditional teaching mode and multimedia network-assisted teaching
2	Grasp the “degree” of using multimedia network-assisted teaching
3	Teachers play an active guiding role to create a Japanese teaching situation
4	Establish and improve the network implementation platform for basic Japanese teaching

**Table 3:** Teachers play an active guiding role to create a Japanese teaching situation.

1	Teachers should guide students to clarify learning goals, learning methods, etc., and develop good study habits.

2	When using multimedia networks to assist teaching, teachers should give full play to the dominant advantages of teachers in traditional teaching, give appropriate explanations in the process of playing the courseware, and create “dialogue” and “cooperative” by setting up questions and answers, discussions, etc. Teaching scenarios, guide students to actively participate in the learning process of using multimedia network-assisted teaching, and give full play to students' learning initiative

3	Teachers should guide students to use multimedia technology and network resources correctly and reasonably. In view of the chaos of online Japanese materials, teachers can recommend reliable Japanese learning websites, Japanese newspapers, Japanese learning software, Japanese corpora, etc. to students, so as to provide students with effective learning materials

4	Teachers can teach students efficient retrieval, analysis, and sorting methods, guide students to choose appropriate learning content, and improve learning efficiency.

## Data Availability

The labeled data set used to support the findings of this study is available from the corresponding author upon request.
